# Production of Potent Antimicrobial Compounds from *Streptomyces cyaneofuscatus* Associated with Fresh Water Sediment

**DOI:** 10.3389/fmicb.2017.00068

**Published:** 2017-01-25

**Authors:** Zothanpuia, Ajit K. Passari, Preeti Chandra, Vincent V. Leo, Vineet K. Mishra, Brijesh Kumar, Bhim P. Singh

**Affiliations:** ^1^Molecular Microbiology and Systematics Laboratory, Department of Biotechnology, Mizoram UniversityAizawl, India; ^2^CSIR-Central Drug Research Institute, Sophisticated Analytical Instrument FacilityLucknow, India

**Keywords:** *Streptomyces cyaneofuscatus*, antimicrobial activity, biosynthetic genes, GC-MS, UPLC-ESI-MS/MS

## Abstract

The genus *Streptomyces* under phylum actinobacteria has been recognized as a prolific source for the production of bioactive secondary metabolites. An actinobacterial strain designated as DST103 isolated from a wetland fresh water sediment of Tamdil Lake, Mizoram, Northeast, India was identified as *Streptomyces cyaneofuscatus* (KY287599) using 16SrRNA gene sequencing which shares 99.87% sequence similarity with *Streptomyces cyaneofuscatus* NRRL B-2570**^T^**. The strain showed broad spectrum antimicrobial activities against Gram negative bacteria (*Escherichia coli* MTCC 739 and *Pseudomonas aeruginosa* MTCC 2453), Gram positive bacteria (*Micrococcus luteus* NCIM 2170 and *Staphylococcus aureus* MTCC 96) and yeast pathogen *Candida albicans* MTCC 3017). The methanolic extract of the strain DST103 exhibited highest antimicrobial activity against *E. coli* (IC_50_ = 2.10 μg/mL) and minimum activity against *S. aureus* (IC_50_ = 43.63 μg/mL). Five antibiotics [trimethoprim (18 μg/g), fluconazole (6 μg/g), ketoconazole (18 μg/g), nalidixic acid (135 μg/g), and rifampicin (56 μg/g)] were detected and quantified using ultra-performance liquid chromatography (UPLC-ESI-MS/MS). Further, biosynthetic potential genes [polyketide synthases type II, non-ribosomal peptide synthetases, and aminodeoxyisochorismate synthase (*phz*E)] were also detected in strain DST103 which may possibly be responsible for the production of antimicrobial compounds. Additionally, gas chromatography-mass spectrometry analysis showed the presence of four volatile compounds which might be responsible for their diverse biological activity. The present study revealed the presence of bioactive compounds in strain DST103, which may be a promising resource for the discovery of novel bioactive metabolites against wide range of pathogens.

## Introduction

Microbial secondary metabolites are the organic compounds having potential for the discovery of new drugs to fight against antibiotic resistance (David et al., 2014). They are increasingly required with the emergence and continued persistence of multiple drug resistant (MDR) disease causing microorganisms and still the bacterial infections remain the second leading cause of death worldwide (Procopio et al., 2012). To overcome this, an attempt has been made by various researchers to improve the existing antibiotics or discover the new antibiotics with improved effectiveness (Parungao et al., 2007). Among the microorganisms, phylum Actinobacteria (order - *Actinomycetales*), represent an outstanding and notable source for the production of new bioactive secondary metabolites including antibiotics (Stach et al., 2003; Goodfellow and Fiedler, 2010). The phylum alone is accounting for the production of an approximately 75% of the total bioactive compounds including antibiotics with more than 70% produced by member of the genus *Streptomyces* (Berdy, 2005; Das et al., 2010; Subramani and Aalbersberg, 2012). Genus *Streptomyces* remains prolific producers of novel compounds with a variety of biological activities including antimicrobial, anti-cancer agents and other pharmaceutically useful compounds (Berdy, 2005; Kim et al., 2008; Saurav and Kannabiran, 2012; Wang et al., 2013; Rajan and Kannabiran, 2014; Ser et al., 2015). They are widely distributed in various ecosystems like soils, fresh waters, marine environments and lakes (Goodfellow and Williams, 1983). A continuous screening of potential bacterial taxa for secondary metabolite production is crucial for the discovery of novel compounds (Lazzarini et al., 2000).

Bio-prospecting studies on actinobacteria are mostly confined to the terrestrial and marine ecosystems and less significance has given to fresh water systems (Radhika et al., 2011). However, there are few reports about the presence of actinobacteria from fresh water ecosystems worldwide (Sibanda et al., 2010; Radhika et al., 2011; Saravanan et al., 2015) where they play an important role in carbon cycle and degradation of recalcitrant organic matter (Kuznetsov, 1970). At present, there is a significant decline in discovering novel bioactive compounds from terrestrial actinobacteria (Alvan et al., 2011) which signified the needs to search for biologically active compounds from such alternative sources like fresh water resources.

In recent years, an attempt has been made by many researchers in search of new antibiotics from different unexplored habitats (Mitra et al., 2008; Goodfellow and Fiedler, 2010). Investigation of antimicrobial secondary metabolites producing actinobacteria from various ecosystems of Northeast India is reported by a number of researchers (Talukdar et al., 2012; Sharma et al., 2014, 2016; Passari et al., 2015; Zothanpuia et al., 2015). After literature review, Tamdil, a fresh water lake of Mizoram, North east India, which is one of the 115 wetlands in India has been found unexplored ecosystem for actinobacterial research. Even though this lake was reported earlier (Zothanpuia et al., 2016) as a significant source for bacterial isolation.

In this perspective the present study was carried out that resulted in the selection of a promising *Streptomyces* strain DST103 from the fresh water sediment samples of wetland, Tamdil lake Mizoram, India. The present study is intended to examine the antimicrobial biosynthetic potential of *Streptomyces cyaneofuscatus* against various Gram positive and Gram negative bacterial pathogens, to detect the genes (PKSII, NRPS and *phz*E) responsible for it, to characterize antibiotic production using ultra-performance liquid chromatography (UPLC-ESI-MS/MS) and to determine the volatile compounds by using Gas chromatography-mass spectrometry (GC-MS).

## Materials and Methods

### Sample Collection

Water sediment samples were collected from a wetland, fresh water Tamdil Lake (23° 44′N; 92° 57′E) of Mizoram, India during the month of May 2013. Samples were stored in a sterile screw capped tube and brought into Molecular Microbiology and Systematic Laboratory, Department of Biotechnology, Mizoram University. The samples were preserved at 4°C till it was processed.

### Isolation and Enumeration of Actinobacteria

Actinobacteria were isolated by serial dilution and spread plate technique in eight different media [Starch Casein Agar (SCA), Yeast Extract Malt Extract Agar (ISP2), Actinomycetes Isolation Agar (AIA), Streptomyces Agar (SA), Glycerol Aspargine agar (ISP5), Tyrosine agar medium (ISP7), Tap water Yeast Extract Agar (TWYE), Trypticase soya agar (TSA)]. Serial dilution was performed by preparing stock solution with 1 mL of water sediment sample and 10 ml of sterile distilled water in a test tube and agitated for 10 min. The suspension was serially diluted up to dilutions of 10^-3^ and spread on different media supplemented with cycloheximide (30 μg/ml) to inhibit fungal growth and nalidixic acid (30 μg/ml) to inhibit the growth of Gram negative bacteria. Plates were incubated at 28°C for 14 days and the pure culture of isolates were preserved on 20% glycerol and on their respective slant at 4°C for further studies.

### Phenotypic Characterization of Actinobacterial Isolates

The isolates were characterized after 14 days of incubation at 28°C. The cultural characteristics such as color of aerial and substrate mycelium, characteristics of the colony, color, and morphology of the spore chain and diffusible pigments production were studied (Goodfellow and Haynes, 1984). The purified strains were analyzed and identified as described in the International *Streptomyces* Project (ISP) (Shirling and Gottlieb, 1966). Using oil immersion microscope, the mycelium structures was observed and the organism was identified according to *Bergey’s Manual of Determinative Bacteriology*, 9th edition. The spore chain morphology and ornamentation of the selected potential strain was also analyzed by field emission gun- scanning electron microscope (FEG-SEM) (Passari et al., 2016).

### Evaluation of Antimicrobial Activity of Actinobacterial Isolates

Antimicrobial screening of actinobacterial isolates were performed against five pathogenic bacteria such as Gram positive bacteria, *Staphylococcus aureus* MTCC-96, *Bacillus subtilis* NCIM-2097, and *Micrococcus luteus* NCIM-2170; Gram negative bacteria *viz., Pseudomonas aeruginosa* MTCC-2453, *Escherichia coli* MTCC-739 and *yeast Candida albicans* MTCC-3017. All the pathogens were obtained from Microbial Type Culture Collection (MTCC), Chandigarh, and National Collection of Industrial Microorganisms (NCIM), Pune, India and maintained in the Laboratory. The bacteria and yeast strains were cultured in nutrient agar medium and Sabouraud dextrose medium at 37°C and 25°C, respectively. A single pure colony of actinobacterial isolates were inoculated in tryptone yeast extract broth (ISP1) and incubated at 28°C, 150 rpm for 7–15 days. The grown cultures were centrifuged at 8,000 rpm for 5 min and the supernatant was used for antimicrobial activity by agar well diffusion method (Saadoun and Muhana, 2008). Bacterial pathogens were spread on LB modified agar plate, and 6 mm diameter wells were prepared by using sterile cork borer. In each well, 70 μl clear actinobacteria cell free supernatant was dispensed, and the plates were incubated at 37°C for 24 h. The antimicrobial activities of the isolates were determined by measuring the inhibition zone around each well. All experiments were performed in triplicates and mean was calculated.

### Molecular Identification and Phylogenetic Analysis

#### Genomic DNA Isolation and 16S rRNA Gene Amplification

Genomic DNA of selected strain was extracted using In-vitrogen DNA isolation kit (K182002) following the manufacturer’s protocol. The DNA quantity was checked at 260/280 using spectrophotometer (Thermo scientific Multiskan GO micro plate reader). PCR amplification of 16S rRNA gene was carried out using universal bacterial primers PA (5′- AGAGTTTGATCCTGGCTCAG -3′) as forward primer and PH (5′- AAGGAGGTGATCCAGCCGCA -3′) as reverse primer (Weisburg et al., 1991). Reaction was performed on Veriti thermal cycler (Applied Biosystem, Singapore) in a total volume of 25 μl containing 50 ng of template DNA, 10 pmol of each primer, 2.5 mM of dNTPs, 1X PCR buffer with 1.5 mM MgCl_2_, 1 U/μl of *Taq* DNA polymerase. Reaction was performed under following conditions: initial denaturation at 95°C for 4 min, followed by 30 cycles of denaturation at 94°C for 30 s, annealing at 57.5°C for 40 s and extension at 72°C for 1.3 min with final extension step at 72°C for 10 min. A negative control reaction mixture (without DNA template) was also included with each set of PCR reactions. The amplified PCR product was checked using 1.3% agarose gel electrophoresis using TAE buffer. The PCR bands were analyzed under UV light and documented using a Bio Rad Gel Doc XR^+^ system (Hercules, CA, USA). The PCR products of 16S rRNA gene was purified by quick PCR purification kit (In-vitrogen) and sequencing was done commercially at SciGenome Pvt. Ltd. Cochin, India.

#### Phylogenetic Analysis Based on 16S rRNA Gene Sequences

DNA sequences were compared with the sequences retrieved from NCBI database by using BLASTn search tool (Tamura et al., 2011). Type strains of top fifteen sequences with highest scores were retrieved from EzTaxon database (Kim et al., 2012) and multiple sequence alignment was performed using the Clustal W software packaged in MEGA 6.0 (Thompson et al., 1997). The evolutionary models were selected based on the lowest Bayesian Information Criterion (BIC) scores and highest Akaike Information Criterion (AIC) values using MEGA 6.0 (Saitou and Nei, 1987). Phylogenetic tree was constructed by neighbor joining method using MEGA 6.0 software with Tamura 3 parameters model (*R* = 1.25) (Saitou and Nei, 1987; Tamura et al., 2011), using *E. coli* as an out group. The significance of the branching order was determined by bootstrap analysis of 1000 replicates using *p*-distance model (Felsenstein, 1985). The obtained nucleotide sequence of the 16S rRNA gene of the potential strain was deposited in NCBI GenBank and trees were analyzed and checked using program FigTree 1.3.1.

#### Methanolic Extraction of Potential Isolates and Antimicrobial Assay

The selected isolate was grown in tryptone yeast extract (ISP1) broth at 28°C for 30 days and the culture filtrate was used for the extraction using methanol 1:1 ratio (v/v). Methanol extract was prepared in different concentrations (100, 25, 500, and 1000 μg/ml) with 10% dimethyl sulphoxide (DMSO) and used for antimicrobial activity following agar well diffusion method (Saadoun and Muhana, 2008; Gebreyohannes et al., 2013).

#### Determination of Minimum Inhibitory Concentration (MIC) of Potential Isolates

Minimum inhibitory concentration (MIC) of selected strain was determined by following broth micro dilution technique using 96-well microtiter plate (Eloff, 1998). Crude extract of the selected strain was prepared with 10% DMSO in different concentrations (100, 25, 500, and 1000 μg/ml). The bacterial pathogens were grown up to a final concentration of 1.0 × 10^-4^ CFU/mL (OD = 0.402). Different concentrations of the crude extract were added in 96-well microtiter plate containing a bacterial culture as test and without bacterial culture as controls. Antibiotic (ampicillin, 0.01 μg/ml) along with bacterial cultures were used as positive control, DMSO containing bacterial cultures were used as negative control. The plates were incubated at 37°C for 36 h and absorbance was taken at 620 nm in spectrophotometer UV-VIS (MultiscanTM GO, Thermo Scientific, MA, USA). IC_50_ was expressed as the concentration (μg/ml) of crude extract at which 50% of bacterial growth was inhibited and was calculated using the calibration curve by linear regression.

### Detection of Antibiotics using Ultra-Performance Liquid Chromatography (UPLC-MS/MS)

#### Preparation of Standard Solution

Mixed stock solution containing standard antibiotics (trimethoprim, fluconazole, ketoconazole, nalidixic acid, and rifampicin) were prepared in methanol. Mixed standards were diluted with methanol within the ranges from 0.5 to 500 ng/mL to prepare the working standard solution used for plotting calibration curve. The standard stock and working solutions were all stored at –20°C until use and vortexed prior to injection.

#### Instrumentation and Analytical Conditions

An acquity ultra-performance liquid chromatography (UPLC^TM^) system consisting of autosampler and a binary pump (Waters, Milford, MA, USA) was used for analysis. Compounds were separated using an acquity BEH C18 (2.1 mm × 50 mm, 1.7 μm; Waters, Milford, MA, USA) analytical column. The mobile phase consisted of two solvents: 0.1% (v/v) formic acid in water (A) and acetonitrile (B) with the gradient program performed of a linear increase from 0 to 1 min, 12–90% B; 2–4 min, 90–95% B; 4–5 min, 95–12% B, 1 min post-run and 12% B. The flow rate was set at 0.35 ml/min with injection volume 5 μl. UPLC system coupled to triple-quadrupole linear ion trap mass spectrometer (API 4000 QTRAP^TM^ MS/MS system from AB Sciex, Concord, ON, Canada) having electro spray (Turbo V^TM^) ion source was run in positive and negative ionization mode. The following optimized parameters were used for positive control: ion spray voltage (5500 V); turbo spray temperature (450°C); heater gas (gas 2, 50 psi); nebulizer gas (gas 1, 50 psi); collision gas (medium); curtain gas (20 psi). The mass spectrometric conditions was optimized by injecting 100 to 500 ng/ml solutions of each analytes at 10 μl/min using a Harvard ‘22’ syringe pump (Harvard Apparatus, South Natick, MA, USA). For each compound, highest profusion of precursor-to-product ions was selected for MRM quantitation. Data acquisition and instrument control were done by Analyst (1.5.1 software package, AB Sciex). The spectra enclosed the range from m/z 100 to 1000 for analysis of full scan ESI-MS. Flow injection analysis was used to optimized all the MS parameters for reference analytes such as precursor ion (Q1), product ion (Q3), entrance potential, declustering potential, cell exit potential and collision energy in positive and negative ESI mode. MRM parameters were optimized to attain the most copious, specific and stable MRM transition for every compound (**Table 1**).

**Table 1:** LC-MS/MS optimized parameters for the detection of antibiotics.

Analytes	*rt* (min)	Q1	Q3	Ion species	DP	EP	CE	CXP
Trimethoprim	0.9	291.2	231.2	[M+H]^+^	149	6	33	10
Fluconazole	1.07	307.1	220.1	[M+H]^+^	59	10	27	8
Ketoconazole	1.46	532.1	82	[M+H]^+^	106	10	68	10
Nalidixic acid	1.58	233.1	215.1	[M+H]^+^	49	8	21	8
Rifamycin	1.83	823.5	791.4	[M+H]^+^	53	9	24	19

### Detection and PCR Amplifications of Biosynthetic Gene Fragments (PKSII, NRPS and *phz*E):

The potential antimicrobial isolates were subjected for the amplification of genes for Polyketide synthase type II (PKS II), aminodeoxyisochorismate synthase (*phz*E) and non-ribosomal peptide synthetase (NRPS). The following degenerate primers (**Table 2**) were used for amplification and detection of PKS-II, *phz*E and NRPS gene fragments according to Yuan et al. (2014) with some modifications. The action was carried out in the Veriti thermal cycler (Applied Biosystems, Singapore) under the following conditions.

**Table 2:** Primer sets used for the amplification of secondary metabolite biosynthetic genes.

Gene	Primer	Length (bp)	Reference
PKS II (KS1F, KS1R)	5′-TSGCSTGCTTGGAYGCSATC-3′ 5′-TGGAANCCGCCGAABCCTCT-3′	554	Wawrik et al., 2005
*phz*E (phzEf, phzEr)	5′-GAAGGCGCCAACTTCGTYATCAA-3′ 5′-GCCYTCGATGAAGTACTCGGTGTG-3′	450	Schneemann et al., 2011
NRPS (A3F, A7R)	5′-GCSTACSYSATSTACACSTCSGG-3′ 5′-SASGTCVCCSGTSGCGTAS-3′	700	Ayuso-Sacido and Genilloud, 2005

PKS II (50 μL): 3 μL template, 5 μL 10× buffer, 1 μL MgCl_2_ (25 mM), 1 μL DMSO (10%), 5 μL dNTP (2.5 mM), 1.8 μL each primer (10 μM) and 5 U Taq DNA polymerase; 5 min at 95°C, followed by 35 cycles of 1 min at 95°C, 1 min 30 s at 58°C and 2 min at 72°C, followed by a 10 min extension at 72°C.
NRPS (50 μL): 3 μL template, 5 μL 10× buffer, 1 μL MgCl_2_ (25 mM), 1 μL DMSO (10%), 5 μL dNTP (2.5 mM), 2 μL each primer (10 μM) and 5 U *Taq* DNA polymerase; 5 min at 95°C, followed by 35 cycles of 1 min at 95°C, 2 min at 59°C and 4 min at 72°C, followed by 10 min extension at 72°C.
*phz*E (25 μL): 2 μL template, 2.5 μL 10× buffer with 15 mM MgCl_2_, 2 μL BSA (1 mg/mL), 2 μL dNTP (2.5 mM), 0.8 μL each primer (10 μM) and 2 U Taq DNA polymerase; 4 min at 94°C, followed by 35 cycles of 1 min at 94°C, 1 min at 55°C and 2 min at 72°C, followed by a 8 min extension at 72°C.

A Reaction mixture without DNA template of actinobacteria was also incorporated with each set of PCR as negative control. PCR products were visualized under gel documentation system. The PCR products of PKS II, NRPS and *phz*E were purified and sequenced commercially at Sci Genome Pvt. Ltd. Cochin, India.

### Gas Chromatography Mass Spectroscopy (GC-MS) Analysis of Strain DST103

The chemical compounds present in the selected strain was analyzed and identified using GC-MS as described by Ser et al. (2015) and Sharma et al. (2016) with some modifications. Crude extract of the strain was dissolved in spectroscopy-grade methanol. GC-MS analysis was performed on Perkin Elmer Turbo mass with single quadrupole fitted with PE-5MS column (length 30 m, thickness 0.25 μm, internal diameter 25 mm). The oven temperature was started at 75°C held for 5 min and ramped at 10°C per min up to 280°C and held for 10 min. One microliter of the sample was injected at 250°C using helium as carrier gas, split at the ratio of 1:30. Mass Spectrometer was run in the electron ionization (EI) mode in 220°C at 70 eV with a scan range of 10 to 620 m/z. The peaks were analyzed and identified by matching the mass spectra with the National Institute of Standards and Technology (NIST, USA) library.

### Phylogenetic Analysis Based on Biosynthetic Genes Sequences

Amino acid sequences of PKS type II, NRPS and phzE genes were compared with the sequences obtained from NCBI GenBank with the BLASTp algorithm and aligned using Muscle software packaged in MEGA 6.0 (Edgar, 2004). The evolutionary models were selected based on the lowest Bayesian Information Criterion (BIC) score values using MEGA 6.0 (Saitou and Nei, 1987). All positions containing gaps and missing data were removed from the phylogenetic analysis. Maximum likelihood (ML) phylogenetic tree for PKS type II and NRPS gene were constructed using WAG model whereas Jones Taylor Thomton (JTT model) was used for constructing ML phylogenetic tree for phzE gene (Saitou and Nei, 1987).

### Statistical Analysis

The antimicrobial assay was performed in triplicate process and repeated for three times. Readings was taken as the mean ± standard deviation of mean of three replicates calculated using Microsoft Excel XP 2010. One way analysis of variance (ANOVA) was employed to test the significant differences (*P* ≤ 0.05) between antimicrobial activities of different isolates using SPSS software version 20.0.

## Results

### Isolation and Characterization of Actinobacterial Strains

A total of 50 strains of actinobacteria were isolated from fresh water sediment samples collected from Tamdil Lake of Mizoram, Northeast India. All the obtained isolates were purified and identified based on morphological characteristics after two to three weeks of incubation on different media. Most of the isolates showed strain specific morphological characters such as slow growth, color of mycelia from yellow, brownish white to blackish white, while, some isolates formed brown colored pigments on the media (**Figure 1A**). The field emission gun-scanning electron microscopy (FEG-SEM) analysis revealed that the aerial mycelia produced spore chains that were spiral and long (**Figure 1B**).

**FIGURE 1:** **(A)** Morphological appearance of Strain DST103 on TSA medium after three weeks of incubation; **(B)** field emission gun- scanning electron microscope (FEG-SEM) analysis showing spore chain morphology of Strain DST103; **(C)** Antibacterial activity of Strain DST103 against bacterial pathogen *Bacillus subtilis*.

### Evaluation of Antimicrobial Activity

The isolated actinobacterial isolates were evaluated for their *in vitro* antimicrobial activity against five bacterial pathogens: *S. aureus, M. luteus, B. subtilis, P. aeruginosa, E. coli*, and yeast *C. albicans*. From a total of 50 isolates tested, 10 isolates showed positive antibacterial activity against at least 3 of the tested 6 pathogens (Supplementary Table S-1). The isolate DST103 showed positive activity against 5 tested pathogens, which was indicated by its activity (15 mm inhibition diameter) against *E. coli* followed by *C. albicans* (12.6 mm), *B. subtilis* (11.2 mm), *P. aeruginosa* (8 mm), *S. aureus* (7 mm) and relatively no activity against *M. luteus* (**Table 3**). All the isolates showed positive activity against *E. coli*, while most of the isolates were susceptible to *S. aureus* and *M. luteus*. Isolate DST103 having a broad spectrum antimicrobial activity was selected for further investigations (**Figure 1C**).

**Table 3:** Antimicrobial activity of strain DST103 against selected pathogens.

Strain no.	Antimicrobial activity Zone of inhibition [mean (mm) ± SD]					
	*S. aureus*	*E. coli*	*P. aeruginosa*	*B. Subtilis*	*M. luteus*	*C. albicans*
**DST103**	07.0 ± 0.10	15.0 ± 0.03	08.0 ± 0.25	11.2 ± 0.10	00.00 ± 0.0	12.60 ± 0.05

### Characterization and Phylogenetic Affiliation of Isolate DST103

Selected isolate DST103 was subjected to amplification of partial 16S rRNA gene and the obtained sequence (1404 bp) having an average G+C content of 58.4% was identified as *Streptomyces cyaneofuscatus* (NCBI GenBank accession number KY287599) which shares 99.87% sequence similarity with *Streptomyces cyaneofuscatus* NRRL B-2570**^T^**. The sequence was aligned by the BLAST analysis tool along with the type strains retrieved from EzTaxon databases. Phylogenetic tree was constructed to check the unique molecular taxonomic position of the strain based on neighbor joining method with Tamura 3-parameter model according to lowest BIC values using Mega 6.0. Gaps were treated by pair wise deletion and the estimated Transition/Transversion bias (R) is 1.25. The phylogenetic tree clearly showed that strain DST103 is closely related to *Streptomyces cyaneofuscatus* NRRL B-2570^T^, as they formed a distinct clade under a bootstrap support value of 89%. The 16S rRNA gene sequence analysis demonstrates that strain DST103 was intimately similar to the type strains *Streptomyces setonii* NBRC 13085^T^ (99.85% similarity) followed by *Streptomyces halstedii* NBRC 12783^T^ (99.82%), *Streotomyces flavovirens* NBRC 3716^T^ (99.8%) (**Figure 2**).

**FIGURE 2:** **Phylogenetic tree of *Streptomyces cyaneofuscatus* strain DST103 showing phylogenetic relationships maximum likelihood method with Tamura 3-parameter model with bootstrap value based on 1000 replicates**.

### Determination of MIC of Strain DST103

The crude methanolic extract of strain DST103 exhibited strong antimicrobial activity against Gram positive bacteria, Gram negative bacteria and yeast pathogen. From our results, we observed that the isolate showed highest activity against *E. coli* (5.42 to 15.89 μg/mL) followed by *C. albicans* (4.12 to 12.6 μg/mL), *B. subtilis* (3.96 to 11.2 μg/mL) and *P. aeruginosa* (3.17 to 8.0 μg/mL), respectively. In 96 well plate assay, strain DST103 showed highest MIC values against *E. coli* (EC_50_ = 2.1 μg/mL) whereas, lowest MIC values was recorded against *S. aureus* (EC_50_ = 43.63 μg/mL). Standard known antibiotic ampicillin was used as positive control and 10% DMSO solvent was used as negative control.

### Detection and Quantification of Antibiotics using UPLC-MRM Method

#### Validation of Analytical Method

As per the guidelines of international conference on harmonization (ICH, Q_2_R_1_) by linearity, solution stability, quantifications and limit of detections, precision and recovery, UPLC-MRM method was validated for quantitative analysis.

#### Linearity, Limits of Detection (LOD) and Quantification (LOQ)

A series of concentrations of standard solute ion were prepared for the establishing calibration curves. The peak areas were plotted against the corresponding concentrations to obtain the calibration curves. LOD and LOQ were determined by calibration curve method. LOD and LOQ were calculated by using following equations. LOD = (3.3 × Sy.x)/S; LOQ = (10 × Sy.x)/S (Where, Sy.x is standard deviation of residuals from line; *S* is slope). The results were listed in **Table 4**. All the calibration curves indicated good linearity with correlation coefficients (*r*^2^) from 0.9989 to 0.9999 within the test ranges. The LOD and LOQ for each reference analyte were less than 0.52 ng/mL and 0.78 ng/ml, respectively.

**Table 4:** Validation parameters used for the detection of antibiotics in strain DST103.

Analytes	Regression equation	*r^2^*	Linear range ng/ml	LOD ng/ml	LOQ ng/ml	Precision RSD (%)		Stability	Recovery RSD (%)
						Intra-day (*n* = 6)	Inter-day (*n* = 6)	RSD (*n* = 5)	
Trimethoprim	*y* = 1116.5 × –2399.2	0.9989	1–100	0.52	0.78	1.23	0.99	1.55	1.44
Fluconazole	*y* = 16698 × –980.72	0.9999	0.5–50	0.11	0.42	1.11	0.58	2.45	1.27
Ketoconazole	*y* = 641.95 × –104.06	0.9996	0.5–50	0.13	0.38	1.08	1.03	1.29	1.45
Nalidixic acid	*y* = 55514 × + 9135.4	0.9996	0.5–100	0.18	0.42	0.78	2.01	1.35	1.09
Rifamycin	*y* = 7410.9 × –5216.3	0.9995	0.5–50	0.10	0.36	0.81	1.67	0.79	0.96

#### Precision, Solution stability, and Recovery

Relative standard deviation (RSD) was employed for precision evaluation. Analytes were determined in six replicates on a single day and by duplicating the experiments over three consecutive days to evaluate intra-day and inter-day variations. The overall precision was not more than 2.01%. Sample solutions stability kept at room temperature was measured at 0, 2, 4, 8, 12, and 24 h by replicate injections. The stability RSD value of analytes is ≤2.45%. Recovery test was applied to evaluate the accuracy by spiking high, middle and lower concentration level of the analytical standards into the samples. Experiments were performed in triplicates at each level. The overall recovery of analytical method developed is in the range of 97.98%–102.12% (RSD ≤ 1.45%) for all analytes which signifies a good accuracy (**Table 4**).

### Quantitative Analysis

In this study UPLC-ESI-MS/MS method was used to quantify five standard antibiotics, i.e., trimethoprim, fluconazole, ketoconazole, nalidixic acid, and rifampicin in isolate DST103. Antibiotics like Nalidixic acid (135.0 μg/g) were present in highest amount followed by rifamycin (56.0 μg/g), ketoconazole (18.0 μg/g), trimethoprim (18.0 μg/g) while fluconazole (6.0 μg/g) was lowest among all. MS spectra and MRM extracted ion chromatogram of five standards and strain DST103 was shown in **Figures 3** and **4**, respectively.

**FIGURE 3:** **MS/MS Spectra of reference analytes; (A)** trimethoprim, **(B)** fluconazole, **(C)** ketoconazole, **(D)** nalidixic acid, **(E)** rifampicin.

**FIGURE 4:** **MRM extracted ion chromatogram of reference analyte: (A)** trimethoprim, **(B)** fluconazole, **(C)** ketoconazole, **(D)** nalidixic acid, **(E)** rifampicin.

### GC-MS Analysis of DST103 Strain

Methanolic extract of strain DST103 was analyzed using GC-MS and identified four volatile compounds by comparison of their mass spectra with the NIST library based on their molecular weight, molecular formula, and retention time. The four compounds were (1) 2-propen-1-amine, n-2-propenyl-; (2) 2-propenal, 3-(1-aziridinyl)-3-(dimethylamino)-; (3) 2-decene, 3-methyl-, (z)-; (4) 5-pyrrolidino-2-pyrrolidone (**Table 5**). The peak area is directly proportional to the amount of compound present in the sample.

**Table 5:** Chemical compounds detected in strain DST103 by GC-MS analysis.

Sl No.	Compound name	Retention time (min)	Area (%)	Formula	Molecular weight (MW)	Quality (%)	Activity	Reference
1	2-propen-1-amine, *n*-2-propenyl-	17.545	8	C_6_H_11_N	97	71	Antibacterial	Senbagam et al., 2016
2	2-propenal, 3-(1-aziridinyl)-3-(dimethylamino)-	17.820	8.96	C_7_H_12_ON_2_	140	76	Antimicrobial	Sheoran et al., 2015
3	2-decene, 3-methyl-, (z)-	18.995	30.00	C_11_H_22_	154	78	Antimicrobial	Kalaiselvan et al., 2012; Idramsa et al., 2016
4	5-pyrrolidino-2-pyrrolidone	19.991	28.03	C_8_H_14_ON_2_	154.209	74	–	–

### Detection of PKS II, NRPS, and *phz*E Gene in DST103 Strain

Biosynthetic potential genes encoding PKS type II, NRPS and aminodeoxyisochorismate synthase (*phz*E) were detected in DST103 strain, which may be responsible for the production of antimicrobial compounds. All the genes were sequenced and sequences were deposited in GenBank accession number (KX595189 for PKSII, KX595190 for NRPS and KX894555 for *phz*E). PCR amplifications using degenerate primers showed the expected bands size of 600, 700, and 400 bp for PKSII, NRPS and *phz*E genes, respectively (**Figure 5**).

**FIGURE 5:** **Detection of antimicrobial biosynthetic genes in strain DST103 (A)** polyketide synthases (PKS) type II; **(B)** Non-ribosomal peptide synthetases (NRPS); **(C)** Aminodeoxyisochorismate (*phz*E) synthase.

### Phylogenetic Analysis Based on Biosynthetic Genes Sequences

BLASTp analysis of the amino acid biosynthetic genes (PKSII, NRPS, and phzE) of strain DST103 revealed 63 to 100% identity with known type strains in the NCBI database. The maximum likelihood phylogenetic tree was constructed using the amino acid sequences of PKS type II gene showed that the strain DST103 was closely related to *Streptomyces* sp. SCAU5110 PKS type II (with sequence similarity of 78%) and *Streptomyces carnosus* (ALP32528) PKS with bootstrap value of 64%. In case of NRPS gene the strain DST103 was clustered with *Streptomyces* sp. 10-28-3A (BAH68821) with sequence similarity of 63% and *Streptomyces lavendulae* subsp. *lavendulae* (BAH68484) with sequence similarity of 61 with 77% of bootstrap supported values, respectively. The *phzE* gene sequences of strain DST103 was 100% identical with *Streptomyces* sp. HB291 (**Figure 6**).

**FIGURE 6:** **Maximum likelihood (ML) phylogenetic tree constructed using amino acid sequences based on WAG model for PKS type II gene (A)** and NRPS gene **(B)** and JTT model for *phz*E gene **(C)**. The scale bar represents the amino acid changes.

## Discussion

Secondary metabolites mainly new and novel antibiotics are in great demand with the increase in multi-drug resistant pathogens. A total of 50 actinobacteria were recovered in the present study using seven different media and among the media employed, SCA proved to be the best medium for isolation of fresh water actinobacteria supported by the findings of Rifaat (2003), Radhika et al. (2011), Zothanpuia et al. (2015). Preliminary screening of the isolates for their antimicrobial activities led to the selection of potential strain DST103 having strong activity against almost all the tested pathogens. The nature of colony of the strain was observed with hard and rough velvety texture on solid media with faint diffusible pigment. The strain showed optimum growth at 28°C on AIA, TSA, and SCA media. A slow growth was also observed on ISP2, AIA, SA, ISP5, and ISP7 media except TWYE medium which was also reported earlier by Passari et al. (2015).

Methanolic extract of the strain showed broad spectrum antimicrobial activity in secondary screening by agar well diffusion method which is in agreement with the finding of Gebreyohannes et al. (2013). It also exhibited good activity in 96 well plates inhibited the growth of pathogenic bacteria (*E. coli, S. aureus, P. aeruginosa*, and *B. subtilis*) and yeast pathogen *C. albicans* responsible for different food borne diseases. Strain DST103 showed positive activity against *B. subtilis* and *P. aeruginosa* with MIC values ranging from 3.96 to 11.2 and 3.17 to 8.0 μg/mL, respectively. The strain DST103 exhibited highest antibacterial activity against *E. coli* (5.42 to 15.89 μg/mL). Similar studies were reported by other researchers as well (Mukai et al., 2009; Kavitha et al., 2010; Atta, 2015; Sharma et al., 2016). This result showed that bioactive compounds having antimicrobial activities were extracellular and could be isolated and quantified that may help in the discovery of new drug (Passari et al., 2015). To best of our knowledge, this is the first report of *S. cyaneofuscatus* having strong antimicrobial activity against bacteria and yeast pathogens.

Results from 16S rRNA gene sequence and phylogenetic analyses revealed that the strain having strong antimicrobial properties was identified as *Streptomyces cyaneofuscatus* strain DST103 which was closely related to *Streptomyces cyaneofuscatus* NRRL B-2570^T^ with 99.87% sequence similarity. This is in agreement with results obtained by Hamedi and Papiran (2015). *Streptomyces cyaneofuscatus* M-27 having antitumor and anti-inflammatory compounds was also isolated from the Central Cantabrian Sea (Afredo et al., 2014).

The antibiotics content of the strain DST103 was quantified using UPLC-ESI-MS/MS method using five standard antibiotics, i.e., trimethoprim, fluconazole, ketoconazole, nalidixic acid and rifampicin. All the five antibiotics used in the study were detected and quantified, antibiotics like nalidixic acid and rifamycin were present with 135.0 and 56.0 μg/g respectively. This finding was similarly reported recently (Passari et al., 2016) that nalidixic acid and rifampicin was quantified with 0.951 and 0.017 mg/g, respectively. The antibiotics content of the strain needs to be checked with more standard antibiotics for further investigation.

Gas chromatography-mass spectrometry is one of the most reliable techniques to identify the constituents of volatile compounds which were employed by a number of researchers (Jog et al., 2014; Tan et al., 2015; Sharma et al., 2016). The GC-MS chromatogram of the strain DST103 crude extract showed four major peaks with different retention time. Four volatile compounds were identified that were grouped into amine, ketones, aldehyde, and alkenes, which were renowned to have antimicrobial properties. Among them 2-decene, 3-methyl-, (z)- an alkene group was detected in highest amount which alone constituted 30% of the total constituents present in DST103 which was also reported to have antimicrobial properties (Kalaiselvan et al., 2012; Idramsa et al., 2016). Other compounds like 2-propen-1-amine, *n*-2-propenyl- an amino group was also detected in strain DST103 which was reported to have antibacterial activity by Senbagam et al. (2016). 2-propenal, 3-(1-aziridinyl)-3-(dimethylamino)- an aldehyde group was also detected and reported to have antimicrobial properties (Sheoran et al., 2015) but no reports has been found on 5-pyrrolidino-2-pyrrolidone as an antimicrobial agent. The significance of this finding is that to best of our knowledge, all the above mentioned compounds have been detected for the first time from *Streptomyces cyaneofuscatus* or even from the phylum actinobacteria.

PCR detection and amplification of biosynthetic genes was crucial for assessing the biosynthetic potential of both culturable and non-culturable microorganisms (Minowa et al., 2007). NRPS, PKS, and *phz*E are biosynthetic systems responsible for the synthesis of a large number of biologically active compounds in actinobacteria and other microorganisms. NRPS and PKS are involved in the synthesis of bioactive peptides and polyketides and *phz*E is involved in the synthesis of the antibiotic, phenazine, playing vital roles in biological control (Ayuso-Sacido and Genilloud, 2005; Yuan et al., 2014). In this study, NRPS, PKS II, and *phz*E gene sequences were detected in DST103 and amplified with the expected size which might be responsible for the regulation of its antimicrobial activity.

The present study revealed the presence of bioactive compounds in strain DST103, which could be a promising source for the discovery of novel bioactive metabolites against wide range of pathogens.

## Author Contributions

ZP: Complete the entire experiments and prepared the draft manuscript. AP, VL, and VM: Supported ZP to fulfill the experiment and also help in preparing the manuscript. PC, BK: conducted HPLC analysis. BS: Experiment checked carefully, verified, and approved the final manuscript.

## Conflict of Interest Statement

The authors declare that the research was conducted in the absence of any commercial or financial relationships that could be construed as a potential conflict of interest.

## References

[B1] AfredoF. B.FiedlerH. P.NavaH.GonzálezV.Sarmiento-VizcaínoA.MolinaA. (2014). Two *Streptomyces* species producing antibiotic, antitumor, and anti-inflammatory compounds are widespread among intertidal macroalgae and deep-sea coral reef invertebrates from the central Cantabrian Sea. *Microb. Ecol.* 69 512–524. 10.1007/s00248-014-0508-025319239

[B2] AlvanG.EdlundC.HeddiniA. (2011). The global need for effective antibiotics - A summary of plenary presentations. *Drug Resis. Updat.* 14 70–76. 10.1016/j.drup.2011.01.00721440487

[B3] AttaH. M. (2015). Biochemical studies on antibiotic production from *Streptomyces* sp.: taxonomy, fermentation, isolation and biological properties. *J. Saudi Chem. Soc.* 19 12–22. 10.1016/j.jscs.2011.12.011

[B4] Ayuso-SacidoA.GenilloudO. (2005). New PCR primers for the screening of NRPS and PKS-I systems in actinomycetes: detection and distribution of these biosynthetic gene sequences in major taxonomic groups. *Microb. Ecol.* 49 10–24. 10.1007/s00248-004-0249-615614464

[B5] BerdyJ. (2005). Bioactive microbial metabolites. *J. Antibiot.* 58 1–26. 10.1038/ja.2005.115813176

[B6] DasS.WardL. R.BurkeC. (2010). Screening of marine *Streptomyces* spp. for potential use as probiotics in aquaculture. *Aquaculture* 305 32–41. 10.1016/j.aquaculture.2010.04.001

[B7] DavidB.WolfenderJ. L.DiasD. A. (2014). The pharmaceutical industry and natural products: historical status and new trends. *Phytochem. Rev.* 14 299–315.

[B8] EdgarR. C. (2004). MUSCLE: multiple sequence alignment with high accuracy and high throughput. *Nucleic. Acids Res.* 32 1792–1797. 10.1093/nar/gkh34015034147PMC390337

[B9] EloffJ. N. (1998). Which extractant should be used for the screening and isolation of antimicrobial components from plants. *J. Ethnopharmacol.* 60 1–8. 10.1016/S0378-8741(97)00123-29533426

[B10] FelsensteinJ. (1985). Confidence limits of phylogenies: an approach using the bootstrap. *Evolution* 39 783–791. 10.2307/240867828561359

[B11] GebreyohannesG.MogesF.SahileS.RajaN. (2013). Isolation and characterization of potential antibiotic producing actinomycetes from water and sediments of Lake Tana. Ethiopia. *Asian Pac. J. Trop. Biomed.* 3 426–435. 10.1016/S2221-1691(13)60092-123730554PMC3644569

[B12] GoodfellowM.FiedlerH. P. (2010). A guide to successfuoprospecting: informed by actinobacterial systematics. *Antonie Van Leeuwenhoek* 98 119–142. 10.1007/s10482-010-9460-220582471

[B13] GoodfellowM.HaynesJ. A. (1984). “Actinomycetes in marine sediments,” in *Biological, Biochemical, and Biomedical Aspects of Actinomycetes* eds Ortiz-OrtizL.BojalilL. F.YakoleffV. (New York, NY: Academic Press) 453–472.

[B14] GoodfellowM.WilliamsS. T. (1983). Ecology of actinomycetes. *Annu. Rev. Microbiol.* 37 189–216. 10.1146/annurev.mi.37.100183.0012016357051

[B15] HamediJ.PapiranR. (2015). Molecular characterization and periplasmic expression of the nlp gene of *Streptomyces cyaneofuscatus* UTMC 2101 in *Escherichia coli*. *Ann. Microbiol.* 65 2047–2052. 10.1007/s13213-015-1043-z

[B16] IdramsaE.SutariningsihS.LaurentiusH. N.RarastoetiP. (2016). Antimicrobial activities of endophytic bacteria isolated from *Cotylelobium melanoxylon* (hook.f.) pierre. *Int. J. Pharm. Bio. Sci.* 7 666–672.

[B17] JogR.PandyaM.NareshkumarG.RajkumarS. (2014). Mechanism of phosphate solubilisation and antifungal activity of *Streptomyces* spp. Isolated from wheat roots and rhizosphere and their application in improving plant growth. *Microbiology* 160 778–788. 10.1099/mic.0.074146-024430493

[B18] KalaiselvanA.GokulakrishnanK.AnandT. (2012). Gas chromatography-mass spectrum analysis of bioactive components of the ethanol extract of *Andrographis paniculata*. *J. Pharm. Biomed. Sci.* 20.

[B19] KavithaA.PrabhakarP.NarasimhuluM.VijayalakshmiM.VenkateswarluY.RaoK. V. (2010). Isolation, characterization and biological evaluation of bioactive metabolites from *Nocardia levis* MK-VL-113. *Microbiol. Res.* 165 199–210. 10.1016/j.micres.2009.05.00219577444

[B20] KimK. J.KimM. A.JungJ. H. (2008). Antitumor and antioxidant activity of protocatechu aldehyde produced from *Streptomyces lincolnensis* M-20. *Arch. Pharm. Res.* 31 1572–1577. 10.1007/s12272-001-2153-719099226

[B21] KimT. U.ChoS. H.HanJ. H.ShinY. M.LeeH. B.KimS. B. (2012). Diversity and physiological properties of root endophytic actinobacteria in native herbaceous plants of Korea. *J. Microbiol.* 50 50–57. 10.1007/s12275-012-1417-x22367937

[B22] KuznetsovS. I. (1970). *Microflora of Lakes and its Geochemical Activity.* Leningrad: Nauka.

[B23] LazzariniA.CavalettiL.ToppoG.MarinelliF. (2000). Rare genera of actinomycetes as potential producers of new antibiotics. *Antonie Van Leeuwenhoek* 78 399–405. 10.1023/A:101028760055711386363

[B24] MinowaY.ArakiM.KanehisaM. (2007). Comprehensive analysis of distinctive polyketide and nonribosomal peptide structural motifs encoded in microbial genomes. *J. Mol. Biol.* 368 1500–1517. 10.1016/j.jmb.2007.02.09917400247

[B25] MitraA.SantraS. C.MukherjeeJ. (2008). Distribution of actinomycetes, their antagonistic behaviour and the physico chemical characteristics of the world’s largest tidal mangrove forest. *Appl. Microbiol. Biotechnol.* 80 685–695. 10.1007/s00253-008-1626-818679673

[B26] MukaiA.FukaiT.HoshinoY.YazawaK.HaradaK.MikamiY. (2009). Nocardithiocin, a novel thiopeptide antibiotic, produced by pathogenic *Nocardia pseudobrasiliensis* IFM 0757. *J. Antibiot.* 62 613–619. 10.1038/ja.2009.9019745839

[B27] ParungaoM. M.MacedaE. B. G.VillanoM. A. F. (2007). Screening of antibiotic producing actinomycetes from marine, brackish and terrestrial sediment of Samal Island, Philippines. *J. Res. Sci. Comput. Eng.* 4 29–38.

[B28] PassariA. K.ChandraP.ZothanpuiaMishraV. K.LeoV. V.GuptaV. K. (2016). Detection of biosynthetic gene and phytohormone production by endophytic actinobacteria associated with *Solanum lycopersicum* and their plant growth-promoting effect. *Res. Microbiol.* 167 692–705. 10.1016/j.resmic.2016.07.00127421813

[B29] PassariA. K.MishraV. K.SaikiaR.GuptaV. K.SinghB. P. (2015). Isolation, abundance and phylogenetic affiliation of endophytic actinomycetes associated with medicinal plants and screening for their in vitro antimicrobial biosynthetic potential. *Front. Microbiol.* 6:273 10.3389/fmicb.2015.00273PMC438800225904906

[B30] ProcopioR. E.DeL.Da SilvaI. R.MartinsM. K.De AzevedoJ. C.De AraujoJ. M. (2012). Antibiotics produced by *Streptomyces*. *Braz. J. Infect. Dis.* 16 466–471. 10.1016/j.bjid.2012.08.01422975171

[B31] RadhikaS.BharathiS.RadhakrishnanM.BalagurunathanV. (2011). Bioprospecting of fresh water actinobacteria: isolation, antagonistic potential and characterization of selected isolates. *J. Pharm. Res.* 4 2584–2586.

[B32] RajanB. M.KannabiranK. (2014). Extraction and identification of antibacterial secondary metabolites from marine *Streptomyces* sp. VITBRK2. *Int. J. Mol. Cell. Med.* 3 130–137.25317399PMC4170486

[B33] RifaatH. M. (2003). The biodiversity of actinomycetes in the river nile exhibiting antifungal activity. *J. Mediterr. Ecol.* 4 5–7.

[B34] SaadounI.MuhanaA. (2008). Optimal production conditions, extraction, partial purification and characterization of inhibitory compound(s) produced by *Streptomyces* Ds-104 isolate against multi-drug resistant *Candida albicans*. *Curr. Trends Biotechnol. Pharm.* 2 402–420.

[B35] SaitouN.NeiM. (1987). The neighbor-joining method: a new method for reconstructing phylogenetic trees. *Mol. Biol. Evol.* 4 406–425.344701510.1093/oxfordjournals.molbev.a040454

[B36] SaravananS.SivakamiR.PremG. K. (2015). Actinomycetes diversity in five fresh water systems of Pudukkottai, Tamilnadu and their antimicrobial activity. *Int. J. Curr. Microbiol. App. Sci.* 4 672–677.

[B37] SauravK.KannabiranK. (2012). Cytotoxicity and antioxidant activity of 5-(2 4-dimethylbenzyl)pyrrolidin-2-one extracted from marine *Streptomyces* VITSVK5 spp. Saudi. *J. Biol. Sci.* 19 81–86. 10.1016/j.sjbs.2011.07.003PMC373055723961165

[B38] SchneemannI.WieseJ.KunzA. L.ImhoffJ. F. (2011). Genetic approach for the fast discovery of phenazine producing bacteria. *Mar. Drugs* 9 772–789. 10.3390/md905077221673888PMC3111181

[B39] SenbagamD.SenthilkumarB.AmuthaR. A.NagarajanG.KalandarA. (2016). *Phytotherapeutic Control of Foodborne Pathogens by Jasminum sambac L. Flowers. The Authors Published by Innovare Academic Sciences Pvt Ltd.* Available at: http://creativecommons.org/licenses/by/4.0/

[B40] SerH.MutalibA. B.YinN.ChanK.GohB.LeeL. (2015). Evaluation of antioxidative and cytotoxic activities of *Streptomyces* pluripotens MUSC 137 isolated from mangrove soil in Malaysia. *Front. Microbiol.* 6:1398 10.3389/fmicb.2015.01398PMC467992626733951

[B41] SharmaP.DasR.KalitaM. C.ThakurD. (2014). Investigation of extracellular antifungal proteinaceous compound produced by *Streptomyces* sp. 5K10. *Afr. J. Microbiol. Res.* 8 986–993. 10.5897/AJMR2013.6264

[B42] SharmaP.KalitaM. C.ThakurD. (2016). Broad spectrum antimicrobial activity of forest derived soil actinomycete, *Nocardia* sp. PB-52. *Front. Microbiol.* 7:347 10.3389/fmicb.2016.00347PMC479659227047463

[B43] SheoranN.AgishaV. N.VibhutiM.AditiK.KesavanS.VibinaV. (2015). Genetic analysis of plant endophytic *Pseudomonas* putida BP25 and chemo-profiling of its antimicrobial volatile organic compounds. *Microbiol. Res.* 173 66–78. 10.1016/j.micres.2015.02.00125801973

[B44] ShirlingE. B.GottliebD. (1966). Methods for characterization of *Streptomyces* species. *Int. J. Syst. Bacteriol.* 16 313–340. 10.1099/00207713-16-3-313

[B45] SibandaT.MabinyaL. V.MazombaN.AkinpeluD. A.BernardK.OlaniranA. O. (2010). Antibiotic producing potentials of three freshwater actinomycetes isolated from the eastern cape province of South Africa. *Int. J. Mol. Sci.* 11 2612–2623. 10.3390/ijms1107261220717525PMC2920555

[B46] StachJ. E. M.MaldonadoL. A.WardA. C.GoodfellowM.BullA. T. (2003). New primers specific for actinobacteria: application to marine and terrestrial environments. *Environ. Microbiol.* 5 828–841. 10.1046/j.1462-2920.2003.00483.x14510836

[B47] SubramaniR.AalbersbergW. (2012). Marine Actinomycetes: an ongoing source of novel bioactive metabolites. *Microbiol. Res.* 167 571–580. 10.1016/j.micres.2012.06.00522796410

[B48] TalukdarM.DuarahA.TalukdarS.GohainM. B.DebnathR.YadavA. (2012). Bioprospecting *Micromonospora* from Kaziranga National Park of India and their anti-infective potential. *World J. Microbiol. Biotechnol.* 28 2703–2712. 10.1007/s11274-012-1080-822806196

[B49] TamuraK.PetersonD.PetersonN.StecherG.NeiM.KumarS. (2011). MEGA5: molecular evolutionary genetics analysis using maximum likelihood, evolutionary distance, and maximum parsimony methods. *Mol. Biol. Evol.* 28 2731–2739. 10.1093/molbev/msr12121546353PMC3203626

[B50] TanL. T. H.SerH. L.YinW. F.ChanK. G.LeeL. H.GohB. H. (2015). Investigation of antioxidative and anticancer potentials of *Streptomyces* sp. MUM256 isolated from Malaysia mangrove soil. *Front. Microbiol.* 6:1316 10.3389/fmicb.2015.01316PMC465991126635777

[B51] ThompsonJ. D.GibsonT. J.PlewniakF.JeanmouginF.HigginsD. G. (1997). The Clustal X windows interface: flexible strategies for multiple sequence alignment aided by quality analysis tools. *Nucleic Acids Res.* 24 4876–4882. 10.1093/nar/25.24.4876PMC1471489396791

[B52] WangC.WangZ.QiaoX.LiZ.LiF.ChenM. (2013). Antifungal activity of volatile organic compounds from *Streptomyces alboflavus* TD-1. *FEMS Microbiol. Lett.* 341 45–51. 10.1111/1574-6968.1208823351181

[B53] WawrikB.KerkhofL.ZylstraG. J.KukorJ. J. (2005). Identification of unique type II polyketide synthase genes in soil. *Appl. Environ. Microbiol.* 71 2232–2238. 10.1128/AEM.71.5.2232-2238.200515870305PMC1087561

[B54] WeisburgW. G.BarnsS. M.PelletierD. A.LaneD. J. (1991). 16S ribosomal DNA amplification for phylogenetic study. *J. Bacteriol.* 173 697–703. 10.1128/jb.173.2.697-703.19911987160PMC207061

[B55] YuanM.YuY.LiH. R.DongN.ZhangX. H. (2014). Phylogenetic diversity and biological activity of actinobacteria isolated from the Chukchi Self marine sediments in the Arctic Ocean. *Mar. Drugs* 12 1281 10.3390/md12031281PMC396721024663116

[B56] ZothanpuiaP.PassariA.SinghB. P. (2015). Molecular characterization of actinomycetes isolated from Tuichang river and their biosynthetic potential. *Sci. Vis.* 15:136.

[B57] ZothanpuiaPassariA. K.GuptaV. K.SinghB. P. (2016). Detection of antibiotic-resistant bacteria endowed with antimicrobial activity from a freshwater lake and their phylogenetic affiliation. *Peer J.* 4:e2103 10.7717/peerj.2103PMC490667227330861

